The article "Regulation of lubricin for functional cartilage tissue regeneration: a review" was published in 2018. Journal: Biomater Res.

# Regulation of lubricin for functional cartilage tissue regeneration: a review

**DOI:** 10.1186/s40824-018-0118-x

**Published:** 2018-03-16

**Authors:** Yunsup Lee, Jaehoon Choi, Nathaniel S. Hwang

**Affiliations:** 1 School of Chemical and Biological Engineering, Institute of Chemical Processes, Seoul National University, 1 Gwanak-ro, Gwanak-gu, Seoul, 151-742 Republic of Korea; 2 Interdisciplinary Program in Bioengineering, Seoul National University, Seoul, 152-742 Republic of Korea; 3 N-Bio/BioMAX Institute, Seoul National University, Seoul, 152-742 Republic of Korea

**Keywords:** Lubricin, Articular cartilage, ECM, Tissue engineering, Superficial zone protein (SZP)

## Abstract

**Background:**

Lubricin is chondrocyte-secreted glycoprotein that primarily conducts boundary lubrication between joint surfaces. Besides its cytoprotective function and extracellular matrix (ECM) attachment, lubricin is recommended as a novel biotherapeutic protein that restore functional articular cartilage. Likewise, malfunction of lubrication in damaged articular cartilage caused by complex and multifaceted matter is a major concern in the field of cartilage tissue engineering.

**Main body:**

Although a noticeable progress has been made toward cartilage tissue regeneration through numerous approaches such as autologous chondrocyte implantation, osteochondral grafts, and microfracture technique, the functionality of engineered cartilage is a challenge for complete reconstruction of cartilage. Thus, delicate modulation of lubricin along with cell/scaffold application will expand the research on cartilage tissue engineering.

**Conclusion:**

In this review, we will discuss the empirical analysis of lubricin from fundamental interpretation to the practical design of gene expression regulation.

## Background

Hyaline cartilage, a typical structure of cartilage in our body, plays a critical role in reducing friction and maintaining a wear-resistant property of articulating joint [1]. However, hyaline cartilage is easily damaged due to various causes such as injuries by repeated stress loading and degenerative joint diseases by natural aging or inflammatory activations [2, 3]. Despite the susceptibility of impairment in hyaline cartilage, anatomical architecture that appears to have no vascular and lymphatic systems limits the native cartilage tissue regeneration [3]. Ongoing therapeutic reconstruction of cartilage involves autologous chondrocyte implantation, osteochondral grafts, and microfracture techniques. Even though these treatment options have been applied for cartilage regeneration, these surgical methods still impede cartilage repair regarding organization and functions [4]. Because of these drawbacks, recent studies pay more attention to tissue engineering that seeks cartilage regeneration via incorporation of cells, scaffolds and growth factors [5]. Cartilage tissue engineering has shed a light on the treatment of damaged cartilage with advantageous progress, yet particular improvement in the regeneration of functional tissue is remaining.

Intricate and discrete mechanical properties of articular cartilage arise from its layered framework with different contents. Typically, articular cartilage is comprised of chondrocytes and abundant extracellular matrices (ECMs) that are primarily built up by type II collagen and proteoglycans [6]. Hierarchically, four distinct layers compose articular cartilage, and these four layers are clearly distinguishable from each other by the configuration of collagen fiber and proteoglycans. Progressing from the very uppermost layer to the lowermost layer, just above the bone, the superficial layer has horizontally ordered fibers, the middle layer has disorganized fibers, the deep layer has vertically ordered fibers to the bone surface, and the last calcified layer has few or no alignment but rather mineralized. Contrarily, the amount of proteoglycan is the least in the uppermost superficial layer and rises in a deeper layer. Not only that, depth of layers, ECM composition, and morphology of cells also vary in each layer [7]. The collagen alignments in different layers resulted in a difference of tensile and shear characteristics. However, distribution of proteoglycans in different layers led to compressive feature that differs from each layer. Particularly, the deep layer is 10 ~ 20 times stiffer than the superficial layer [8, 9]. Along with complicated functionality of articular cartilage structure, collagen fiber arrangement restrains the tissue from swelling, whereas proteoglycans that have a negative charge and cartilage tissue with low permeability facilitate swelling of the tissue via water retention [10]. The water retention capability of the tissue is decisive to withstand physical pressure in dynamic loading condition [11]. Cartilage possesses strong load bearing and low frictional coefficient competence due to collagenous network in a combination of proteoglycan structures [12, 13]. There are many studies that demonstrate mechanical and compositional characteristics of native cartilage tissue in general. However, not many have proved elaborate architecture and role of native cartilage raised in cartilage tissue engineering.

One of the key factors for optimal functionality of articular cartilage lies in lubrication that maintains low coefficients of friction of joints. Lubricin is defined as a chondroprotective glycoprotein corresponding to proteoglycan 4 (PRG4), superficial zone protein (SZP), megakaryocyte stimulating factor (MSF) precursor, and camptodactyly-arthropathy-coxa vara-pericarditis (CACP) protein [14–17]. As a crucial synovial fluid component, lubricin is verified to carry its responsibility for antagonizing abnormal cellular adhesion and overgrowth. The fundamental role of lubricin is lubrication of boundary surface of cartilage [18]. Hence, transmutation of lubricin metabolism would conspicuously influence joint performance. In fact, patients who suffer from osteoarthritis (OA), degenerative joint disease, or CACP syndrome, mutation of a proteoglycan4 (PRG4) gene, undergo severe pain due to the progressive wear of cartilage and consequent deficiency of lubricant [17]. Therefore, supplementary lubricin or recombinant lubricin can be a cue to overcome a hurdle that limited functional cartilage tissue engineering. Furthermore, regulating lubricin expression via ECM modulation, growth factors and cytokines addition with comprehensive approach may be another promising solution to unravel the complexity of cartilage remodeling.

In this review, we outline the structural and functional characteristics of lubricin and further examine lubricin-mimetic polymer synthesis. Moreover, lubricin expression governed by ECM manipulation and growth factors or cytokines incorporation was scrutinized. Many attentions on the lubricin synthesis or controllable expression suggest promising perspective in the treatment of functional cartilage impairment regarding lubrication ability.

## Main body

### Structure and functional role of lubricin

Lubricin, a product of the proteoglycan 4 (PRG4) gene, is highly expressed by synoviocytes and superficial zone chondrocytes [18]. Lubricin, generally known as a proteoglycan, is a glycoprotein that functions as a critical boundary lubricant for articular cartilage and normally isolated from synovial fluid [19]. Since lubricin is secreted by not only synoviocytes but superficial zone chondrocytes, it is also called as superficial zone protein (SZP) [18]. Lubricin seems to have no specific structure as long and flexible glycosylated chain with the length of 200 ± 50 nm [19–21]. However, it consists of several protein domains that provide separate biological functions [18]. Center of the chain is a highly glycosylated long region that contributes to the heavy molecular weight of lubricin [16, 18]. This large and mucinous domain, heavily glycosylated protein part with 76 amino acids repeats expressed in high frequency, is mostly composed of GalNAc, Gal, and NeuAc sugar groups where threonine residues are O-linked [19, 21–23]. With abundant negatively charged and highly hydrated sugar groups, this central domain plays a significant role in lubrication due to strong repulsion via steric and hydration forces [18, 23–27]. Also, there are many studies addressing various biological roles of mucin domain-containing proteins that refer to the protection and adhesion of epithelial surfaces [28], the regulation of cell differentiation [29], and the control of cell growth [30].

Non-glycosylated end domain of the protein consists of subdomains similar to two globular proteins: somatomedin-B (SMB) and homeopexin (PEX) [21]. The amino-terminal of the mucin-like domain is linked to SMB-like domains while carboxyl-terminal is linked to PEX-like domain [18]. These two subdomains, also contained in vitronectin, are known to contribute to cell-cell and cell-extracellular matrix (ECM) interactions [21]. For vitronectin, SMB and PEX domains are responsible for regulation of complement and coagulation systems, mediation of extracellular matrix attachment and promotion of cell attachment and proliferation [31–33].

In general, lubricin appears to function as a main boundary lubricant in articular joints [21, 22, 34]. Chang et al. illustrated that the addition of lubricin lowers the coefficient of friction [35]. Moreover, Jay and coworkers investigated chondroprotective characteristic of lubricin by dissipating strain energy from locomotion. Not only that, Jay et al. found the interaction of lubricin with hyaluronic acid (HA) has a significant effect on the function of lubricin diminishing the shear energy by joint gliding [36]. This was also revealed by the study conducted by Chang et al. [27]. Additionally, lubricin prevents protein deposition onto cartilage surface from synovial fluid, controls synovial growth dependent on adhesion, and inhibits synovial cells adhere to cartilage surface, demonstrated by Rhee et al. [18]. Other authors have suggested that lubricin, also known as superficial zone protein (SZP), has potential biological functions such as cell proliferation, cytoprotection, and self-aggregation and matrix binding [14]. In the absence of lubricin, synovial joints would cause dysfunction, which leads to the pathogenesis of cartilage degeneration [37]. On the other hand, besides from all above beneficial properties of lubricin for articular cartilage, a study claimed that lubricin coats the surfaces of damaged cartilage and inhibits integrative repair [38].

### Fabrication of lubricin-mimetic structure

As mentioned above, the molecular structure of lubricin indicates three different domains like heavily glycosylated and, therefore, hydrophilic central part and both side capped with non-glycosylated globular domains. While the central domain mostly contains negatively charged amino acids, the end sides contain positively charged and hydrophobic amino acids [39]. This composition of lubricin shows high similarity to that of mucin proteins [40]. Mucins particularly bind to epithelial surfaces and form a gel-like protective layer (“mucus”) that is built up by molecules physically entangled or covalently linked by forming disulfide bonds between cysteine residues [21, 39].

There are extensively studied synthetic biopolymers mimicking lubricin in structure and functions. It is suggested that the biological functions of lubricins and mucins derive from the similar mechanism of brushes of end-grafted diblock polyelectrolytes, known as charged polymers [41]. When two polyelectrolytes contact each other, they provide a sharp interface with a low degree of brush-brush interpenetration that makes other molecules able to glide through hydration layer where water binds to the outermost part of charged polymer chains [21, 39]. This results in very low friction coefficient, which may refer to excellent tribological property (“superlubricity”) [39, 42, 43] (Fig. 1). However, not only these molecular properties contribute to the boundary lubricating functions. Also, strong and stable integration of the lubricants to the substrate must be preceded to avoid the molecules’ detachment by compression and shear force [39]. Therefore, the structure of lubricin that contains brush-like glycosylated central domain end-grafted with non-glycosylated domains is also called as “bottle-brush” polymer, which gives the unique properties of lubricin [42] (Fig. 2).

**Fig. 1:** Articular cartilage structure with the illustration of collagen fiber orientation [43]

**Fig. 2:** Schematic representations of (**a**) lubricin and (**b-c**) bottle-brush polymers mimicking lubricin [42]

Bottle-brush polymer structure significantly affects lubricin’s lubricating ability, according to biomaterials chemist, Xavier Banquy. Banquy and his colleague have studied to synthesize triblock polymer, as a synthetic lubricant, with the central bottle-brush architecture. The both end blocks were designed to possess strong adhesive characteristics for efficient adsorption to the substrates. This triblock polymer was proved to mimic the natural lubricant, lubricin, structurally and functionally. In brief, the bottle-brush polymer was synthesized by living radical polymerization called “Atom Transfer Radical Polymerization (ATRP)” in combination with postmodification techniques. The bottle-brush polymer is composed of hydrophobic and flexible methyl methacrylate (MMA) backbone supplemented with polyzwitterionic branches of poly (2-methacryloyloxyethyl phosphorylcholine) (PMPC) for better biocompatibility and lubrication [42].

Similarly, another study was conducted about zwitterionic polymer brushes that possess tunable friction and anti-fouling properties. Zwitterionic poly(3-(1-(4-vinylbenzyl)-1H-imidazol-3-ium-3-yl) propane-1-sulfonate) (polyVBIPS) brushes were synthesized and characterized. With elaborated data, polyVBIPS brushes showed super low fouling surfaces and super low friction surfaces at proper ionic conditions [44]. Therefore, polyVBIPS also displays its possibility to be other alternatives for artificial lubricants. Block copolymer consisting of linear positively charged block and uncharged bottle-brush block was developed by the group with Liu. This polymer intended to mimic the structure of bottle-brush polymers present in cartilage surface for improved lubrication [45].

A recent study has examined the hyaluronic acid (HA) chains aggregation with biocompatible hydrogel particles in aqueous solution as biomimetic artificial lubricants [46]. This study showed the potential of HA-hydrogel particle aggregates as biomimetic lubricants since low friction at high load was observed from HA-hydrogel particle aggregates analogous to natural synovial fluid [46]. The effect of HA interacting with other proteins and biopolymers has also been widely investigated. Seror et al. [47] suggested HA-Aggrecan complex act as a boundary lubricant while others explored the synergistic effect of HA with lubricin to reduce friction between the surfaces [48]. Association of two components exists in synovial fluid also demonstrated a synergetic effect for lubrication. Hyaluronan and dipalmitoyl phosphatidylcholine (DPPC) associate each other and form thick layers characterized by low friction coefficients [49]. With little known about HA functions in lubrication, Yu elucidated that HA can act as a boundary lubricant when mechanically or physically trapped. Self-assembled amino-propyl-triethoxy-silane (APTES) layer on mica provides a surface for HA to chemically graft and cross-link. According to the result from the study, comparing free HA and grafted HA, HA grafted to APTES surface indicated the lower coefficient of friction than free HA [50].

Some other studies have focused on the brushes of polyelectrolytes (charged polymers) adsorbed to sliding surfaces exhibited extremely efficient lubrication [41, 51, 52]. Several studies have emphasized strong hydration layers from those polyelectrolytes and proteins as significant lubrication element [53–55]. Liu and colleagues have fabricated hairy polyelectrolyte brushes-grafted thermosensitive microgels as artificial synovial fluid for biomimetic lubrication. They employed negatively charged poly(3-sulfopropyl methacrylate potassium salt) (PSPMK) brushes grafted poly(N-isopropyl acrylamide) (PNIPAAm) microgels [56]. This PSPMK brushes-grafted PNIPAAm microgel provides a structure like a polyelectrolyte that attribute to great hydration lubrication. This study addressed efficient joint lubrication of hairy microgels with high potentials for artificial synovial fluid [56] (Fig. 3).

**Fig. 3:** Effect of synthesized aqueous lubricants on coefficient of friction (COF) with NBrMGs, SB-g-PNIPAAm, and SB-g-NBrMGs (**a**) of different concentration under the normal load of 5 N at 25 °C (**b**) under different loads (**c**) under the normal load of 5 N at different temperature (**d**) schematic diagram illustrating the hydrophilicity/hydrophobicity transition of NBrMGs and SB-g-NBrMGs around the volume phase transition temperature (VPTT) [56]

Liu group also conducted a study with charged polymer brushes but not with grafted microgel but with grafted hollow silica nanoparticles. With the same charged polymer brush PSPMK, silica nanoparticles were cooperated with this polymer that surrounded the nanospheres [57]. Extensively, this group has studied polymer brushes in combination with different scaffolds such as microgel and nanoparticles for biomimetic lubrication and drug release [56, 57]. A recent study indicated modified polymerization for significantly dense and extended poly(2-(methacryloyloxy)ethyl phosphorylcholine) (pMPC) that exhibited enhanced lubricating properties [58]. Engineering lubricin mimetic molecules (mLub) was also attempted utilizing chondroitin sulfate backbone in combination with type II collagen and hyaluronic acid binding peptides. Lubricin mimic was less vulnerable to degradation via enzymes and easily stick to the articular surface reducing friction. mLub interaction with articular surface and synovial fluid constituents have significantly promoted as a result of cooperating type II collagen and hyaluronic acid binding peptides. Therefore, mLub is one of the potent treatments for early osteoarthritis [59].

### ECM control of lubricin expression

Instead of directly mimicking lubricin structure for artificial lubricants, numerous studies explored optimal extracellular matrix composition for enhancement of lubricin expression, ultimately for better articular cartilage regeneration. The decrease of lubricin expression in osteoarthritic (OA) cartilage was observed by encapsulating cells isolated from osteoarthritic cartilage and non-osteoarthritic cartilage. Chondrocytes from each tissue were encapsulated in poly(ethylene glycol) diacrylate (PEGDA) hydrogel and cultured up to 5 weeks to evaluate the level of lubricin expression. It resulted in a significant down-regulation of lubricin in OA cartilage chondrocytes while interestingly this down-regulation was offset after four weeks of culture [60]. However, biosynthesis of lubricin by damaged autologous chondrocytes without any external treatment is very limited.

The role of fibronectin, also a glycoprotein in the superficial zone of cartilage, was investigated and clarified that it binds lubricin and hyaluronan to mica and improves wear resistance via a solid layer of fibronectin and lubricin [61]. Therefore, additional fibronectin to conventional chondrogenic scaffolds can result in upregulated lubricin expression. Additive recombinant human stromal cell-derived factor 1α (rhSDF-1α), potential chondrogenic progenitor cell (CPC) chemoattractant, to fibrin/hyaluronic acid hydrogel was reported to enhance lubricin expression compared to the hydrogel without rhSDF-1α. SDF-1α, chemokine protein, mainly regulates stem cell migration guiding to damaged tissue, in which cells can be involved in tissue regeneration [62]. Other study found peptide-mediated surface coating platform to engage hyaluronic acid (HA) non-covalently. Through this platform, HA that is a natural lubricant relatively abundant in synovial fluid can be actively captured and anchored to the tissue surface [63] or to the polymeric scaffold for tissue engineering and provide effective lubrication.

In addition to external supplementary components, there were several studies with physical and mechanical stimuli for elevating lubricin expression. Chen and coworkers observed that chondrocyte encapsulated agarose hydrogel, named as tissue engineered cartilage (TEC), showed upregulation of PRG4 (lubricin) expression cultured in bioreactor rather than tissue culture plate culture [64]. Moreover, relevant tensile strain to chondrocyte resulted in increased mRNA level of lubricin [65]. Consistently, Ogawa proved that mechanical motion induces PRG4 expression with specific signaling pathway [66]. This result corresponds to 3D scaffold culture of chondrocytes with and without mechanical stimuli. The expression level of lubricin was enhanced with significant surface motion imposition [67]. Grad and colleagues investigated the effect of simple and complex motion patterns on chondrocyte gene expression that showed enhancement of proteoglycan4 (PRG4) expression with the oscillation of ceramic hip ball and scaffold [68]. A recent study reported lubricin expression level regarding cell passage number and the onset of loading. This study divided the experimental group concerning cell passage number and free of loading or under loading. The researchers concluded that lower passage number of chondrocyte has better ability to synthesize lubricin and dynamic loading followed by free-swelling period gave a better environment for lubricin synthesis compared to other culture environments [69].

Applying electromagnetic fields and combined mechanical stimulation on 3D chondrocyte encapsulated construct also revealed to have an effect on lubricin expression enhancement [70]. Furthermore, comparing the chondrogenic expression level of three types of chondrocytes including auricular (AU), articular (AR) and meniscal (ME) chondrocytes, AR and AU encapsulated collagen construct had relevant lubricin stained while ME constructs only showed the trivial amount of stained lubricin [71]. Lohan et al. also examined articular cartilage repair with same polyglycolic acid (PGA) scaffold, but two different cell type such as articular and auricular chondrocytes that concluded auricular chondrocytes are inappropriate cell type for osteochondral defect repair [72]. Zonal chondrocytes from the superficial zone and middle/deep zone were hypothesized to synthesize proteoglycan 4 (PRG4) in a different manner in response to a monolayer or three-dimensional alginate scaffold. This study resulted in different PRG4 secretion rate according to culture environment and cell origin [73].

Matrix molecules such CS and HA critically influenced lubricin expression, according to Coates. Superficial zone chondrocytes expressed up-regulated lubricin level with both CS and HA addition to alginate scaffold while differentiating mesenchymal stem cells (MSCs) expressed down-regulated lubricin level [74]. However, Grogan demonstrated the reverse result with the previous result. This study examined various types of cartilage extracellular matrix molecules regarding the zonal division of cartilage tissue. The expression level of lubricin was mostly decreased regardless of the type of ECM molecules added. 3D scaffold culture of chondrocytes with zone-specific ECM molecules also indicated a reduction of lubricin expression [75]. The porosity of scaffold was also evaluated for lubricin expression. The bilayered scaffold was prepared for cartilage engineering with different pore size and lubricin was expressed throughout the scaffolds without apparent distinction as a result of histological evaluation [76]. Diamond-like carbon (DLC) film was functionalized to exhibit better tribological properties via mussel-inspired catechol adhesive and grafted polymer brushes. This modified DLC film displayed affordable biological lubrication thus providing a prospective biomedical scaffold with effective tribological property [77].

### Growth factor and cytokine control of lubricin expression

The addition of growth factors in the environment of cell culture, as a chemical stimulus, was also examined to elucidate the role of growth factors in lubricin expression. In this part, we discussed various kinds of growth factors and cytokines that showed effect on lubricin synthesis.

The recent study by Schmidt et al. found that transforming growth factor β (TGF-β1) markedly stimulated lubricin secretion by chondrocytes in the surface of articular cartilage, while interleukin (IL)-1α depressed the expression level of lubricin and no effect by insulin-like growth factor 1 (IGF-1) [78]. A similar outcome was observed in the Cheng and colleagues’ study that investigated the expression of PRG4 regulated by either IL-1α or TGF-β1. Chondrocytes isolated from 20-day-old male rats’ condylar cartilage revealed antagonistic effect to the the mRNA expression level of PRG4; reduction by IL-1α and increased by TGF-β1 [79]. Comparably, how different part of the bovine knee joint such as the superficial zone of articular cartilage, synovium, meniscus, and anterior and posterior cruciate ligaments, respond to IL-1β and TGF-β1 was considered. All four explant cultures appeared with significant enhancement of SZP with TGF-β1 and reduction of SZP with IL-1β [80].

More profound consideration of chondrocytes’ ability to secrete lubricin about cytoskeletal modulation was identified. The functional cytoskeleton is one of the decisive factors to lubricin expression induced by TGF-β1. TGFβ-mediated SZP synthesis notably decreased with the pharmacological regulation of actin and microtubule polymerization. The hypothesis of the Rho family GTPases that plays a role in mediating cytoskeleton and lubricin signaling pathway experimented. If small molecular drugs limited the activity of Rho GTPases, SZP synthesis in media via TGF-β1 induction was restrained. Collectively, lubricin accumulation by articular chondrocytes is adjustable by controlling Rho family GTPases, and this suggests a possible technique of lubrication improvement in cartilage tissue engineering [81].

Also, TGF-β/BMP (bone morphogenetic protein) superfamily member showed different regulation of lubricin deposition by superficial zone articular chondrocytes and synoviocytes (Fig. 4). Niikura and colleagues found that both superficial zone articular chondrocytes and synoviocytes were considerably affected by TGF-β. However, synoviocytes were more responsive to BMP family members than were superficial zone articular chondrocytes [82]. Moreover, fibroblast growth factor 2 (FGF-2) and platelet-derived growth factor (PDGF) also facilitated the synthesis of lubricin in monolayer cultures [83]. According to the study conducted by Liu et al. bone-derived mesenchymal stem cells (BMSCs) secreted the highest amount of lubricin when exposed to a combination of all TGF-β1, BMP-7, and ketogenic (KGN), heterocyclic compound, in vitro [84]. In addition to the growth factors, optimal cellular aggregation along with differentiation time has been shown to maximize the lubricin production by differentiating stem cells. During the course of chondrogenic differentiation, MSCs synthesize cartilage related ECMs. According to the study by Musumeci and colleagues, a significant amount of cartilage ECMs, including lubricin, are produced at day 21 of chondrogenic differentiation [85]. In addition, Nakagawa and colleagues have demonstrated that the physical cellular aggregation of MSCs was sufficient to induce lubricin expression both in vitro and in vivo [86].

**Fig. 4:** **a** and **b**, Effects of bone morphogenetic protein (BMP) family members on SZP accumulation in superficial zone articular chondrocytes (**a**) and synoviocytes (**b**). Primary superficial zone articular chondrocytes and synoviocytes were cultured for 3 days as monolayers in serum-free chemically defined medium with or without the addition of BMPs or growth differentiation factor 5 (GDF-5). SZP accumulation in the culture medium was quantified by enzyme-linked immunosorbent assay. Responses to BMPs were much higher in synoviocytes than in chondrocytes. * = *P* < 0.05; ** = *P* < 0.01, versus control. C and D, Effects of concurrent treatment with TGFβ1 (1 ng/ml) and BMPs (100 ng/ml) on SZP accumulation in superficial zone articular chondrocytes (**c**) and synoviocytes (**d**). SZP accumulation with the combined treatment was significantly higher than that observed with each treatment alone (*P* < 0.05), and the additive action was seen in both superficial zone articular chondrocytes and synoviocytes. Values are the mean and SEM from 7 individual experiments, each with cartilage from a different animal. T + B2 = TGFβ1 plus BMP-2; T + B4 = TGFβ1 plus BMP-4; T + B7 = TGFβ1 plus BMP-7; T + G5 = TGFβ1 plus GDF-5 [82]

Cell surface glycosaminoglycans (GAGs), such as heparan sulfate (HS), heparin, and chondroitin sulfate (CS), were proved to have an effect on the TGF-β1 response that activates lubricin synthesis. To be specific, exogenous HS and CS increased lubricin expression level while heparin showed opposite response, hindered lubricin formation [87]. Given its wide scope, cytokines such as Oncostatin M (OSM), IL-1β and tumor necrosis factor (TNF-α) have the potential to control the expression of lubricin as well as growth factors [83, 88]. Lubricin was more synthesized with the inclusion of OSM that presents the capability of lubricin-metabolism modulation. Contrarily, IL-1β and TNF-α down-regulated lubricin level expressed by chondrocytes [88]. Platelet-rich plasma (PRP) consists of numerous autologous growth factors derived from platelets. On top of that, PRP itself includes superficial zone proteins (SZP). Without a precise review of which factor has influenced elevated SZP synthesis by chondrocytes, SZP accumulation by supplementing PRP in culture medium was noted [89].

## Conclusion

The gradual destruction of cartilage owing to multi-factor disorders like osteoarthritis (OA) and CACP syndrome has been persistently examined for the efficient treatment utilizing the field of tissue engineering. Engineering of Articular cartilage has made a reasonable step towards cartilage repair during the last few decades. Some studies have reported potent therapies via direct delivery of chondrocytes to defect site, osteochondral autograft transplantation to the lesion, and surgical microfracture technique. On the other hand, an appropriate function of reconstructed cartilage is remaining question and challengeable issue to overcome. In other respects, the establishment of functionally mature articular cartilage can be achieved by reinforcement of lubricin, lubricating superficial zone protein (SZP). Numerous studies were extensively conducted to examine principle mechanism of lubricin function by its structure. Moreover, experimental attempts to mimic lubricin not only structurally but also functionally were proclaimed. Applying fine or precise tuning of cellular microenvironment using ECM macromolecules, synthetic or natural polymers, growth factors and cytokines was also discussed. Various approaches have done much to the technical advancement of cartilage repair by successfully employing lubricin synthesis and lubricin expression level alteration. Nonetheless, there are some concerns regarding technical difficulties and potential side effects of exogenous variables. Hence, strategies to modulate the lubricin expression for proper functional joint friction reduction would be crucial for successful cartilage tissue formation. As the superficial region of the cartilage is essential for friction reduction, ways to modulate lubricin expression in the superficial zone of articular cartilage would be critical for stable cartilage function.
